# Research on Recognition of Faces with Masks Based on Improved Neural Network

**DOI:** 10.1155/2021/5169292

**Published:** 2021-11-18

**Authors:** Song Zhang, Jiandong Sun, Jie Kang, Shaoqiang Wang

**Affiliations:** ^1^The Affiliated Hospital of Qingdao University, Qingdao 266000, China; ^2^School of Computer and Communication Engineering, China University of Petroleum (East of China), Qingdao 266000, China

## Abstract

**Background:**

At present, the new crown virus is spreading around the world, causing all people in the world to wear masks to prevent the spread of the virus. *Problem*. People with masks have found a lot of trouble for face recognition. Finding a feasible method to recognize faces wearing masks is a problem that needs to be solved urgently.

**Method:**

This paper proposes a mask recognition algorithm based on improved YOLO-V4 neural network and the integrated SE-Net and DenseNet network and introduces deformable convolution.

**Conclusion:**

Compared with other target detection networks, the improved YOLO-V4 neural network used in this paper improves the accuracy of face recognition and detection with masks to a certain extent.

## 1. Introduction

In 2020, the new crown epidemic broke out globally. This sudden epidemic caught countries all over the world by surprise. It not only plunged the global economy into the haze of the Great Recession but also harmed the lives and health of the people in society and brought anxiety and life to life. Although the pandemic has been more than a year now, judging from the current global epidemic situation, the situation is still not optimistic. In the current epidemic situation, the wearing of masks can reduce the chance of infection and has a positive effect on personal protection and global epidemic control.

With the spread of new coronavirus, wearing masks as an effective preventive measure has attracted more and more attention. The behavior of not wearing masks can easily lead to virus transmission, which is not conducive to epidemic prevention and control. In this paper, the target detection network can automatically identify whether travelers wear masks, which is conducive to epidemic prevention and control.

Artificial intelligence has a very wide range of applications in the field of computer vision [1–5] and has achieved excellent results. In [6], the Retina Face detection algorithm is used and the HSV + HOG features of the region are extracted, and SVM is used for training. In [7], a YOLO-Mask algorithm is proposed. The algorithm is based on YOLO-V3, introduces the attention mechanism in the feature extraction network and optimizes the loss function, and then obtains excellent results. In [8], the YOLO-V5 algorithm is improved and then the K-means++ algorithm is used to perform anchor dimensional clustering, determine the anchor parameters, and apply CIoU and diounms to the YOLO-V5 network. In [9], a lightweight network algorithm based on improved YOLO-V4-tiny was proposed, the max module structure was increased to obtain more main features of the target, and the detection accuracy was improved. A bottom-up multiscale fusion was proposed; combining low-level information enriches the feature level of the network, improves feature utilization, and uses CIoU as the frame regression loss function to speed up model convergence. Most of the articles based on mask recognition and face recognition [10–18] use deep learning methods, which have extremely high accuracy.

The best performance of the above algorithms are yoov4 and yoov5 network algorithms. Compared with YOLO-V5, YOLO-V4 has higher accuracy. YOLO-V5 mainly focuses on speed improvement. This article pays more attention to test accuracy, so it is mainly based on the YOLO-V4 network for improvement.

This paper integrates SE-Net and DenseNet networks as the YOLO-V4 reference network and introduces deformable convolution. Compared with other target detection networks, the improved YOLO-V4 network proposed in this paper improves the accuracy of mask detection to a certain extent.

## 2. Method

There are two schemes for mask detection technology. The mainstream scheme is to analyze the pictures in the video surveillance through the target detection model in artificial intelligence and then determine whether the pedestrian is wearing a mask during the surveillance. The second solution is to process the obtained images through traditional image processing methods to determine whether pedestrians are wearing masks during monitoring.

In the mainstream solution, the mask detection system obtains the picture through video surveillance and then normalizes the picture to a uniform size. After inputting it into the model, it detects the face that appears in the picture and locates the face without the mask. The system issues a warning to complete the function of the mask detection system.

A model analysis is generally to input pictures of a fixed size, especially when the model only supports pictures of a fixed size. Generally speaking, high-resolution input can improve the accuracy of model analysis, but high-resolution also means more resource consumption. Therefore, it is generally necessary to make the best choice based on the hardware resources that can be allocated and the performance requirements.

Model selection is generally based on the YOLO-V3 target detection network, using public datasets or your own unique datasets for model training and deployment.

However, video surveillance in mainstream solutions is a real-time video stream, and the system will decompose it into pictures for model analysis. The mainstream solution is based on the efficiency of model analysis and the hardware resources that can be allocated. It is difficult to analyze all the pictures one by one. And some pictures will likely be skipped in the middle.

In the second scheme, the results are obtained by analyzing various traditional image algorithms of monitoring images. Compared with YOLO-V5, YOLO-V4 has higher accuracy. YOLO-V5 mainly focuses on speed improvement. This article pays more attention to test accuracy, so it is mainly based on the YOLO-V4 network for improvement.

In 2020, the YOLO-V4 network turned out, reaching new heights in terms of speed and accuracy. Compared with YOLO-V3, YOLO-V4 has a major change that introduces CSPNet, which makes the skeleton network CSPDarknet-53. Compared with Darknet-53, the CSPDarknet-53 network is only a structural improvement to the original basic module ResUnit. We call the improved basic module CSPUnit.

Compared with ResUnit, the CSPUnit module divides the features in the channel dimension after downsampling. Only half of the features enter the original ResUnit module. After coming out, they are directly spliced with the other half of the features in the channel dimension and finally pass through another convolution operation.

Overall, in terms of accuracy and speed, YOLO-V4 has reached its peak.

## 3. Method Improvement

YOLO-V4 has higher accuracy than YOLO-V5. YOLO-V5 mainly focuses on speed improvement. In this paper, the algorithm pays more attention to the test accuracy, so it is mainly based on the YOLO-V4 network for improvement.

1. Use the classification network DenseNet network and improve it, adding an attention mechanism, and the network model classifies whether pedestrians are passing by
2. The target detection network adopts the YOLO-V4 network, which has high detection accuracy and introduces deformable convolution

The improvement of the DenseNet network in this paper is mainly to add attention mechanism, and the improved topology is shown in Figure 1.

In Figure 1, (a) represents DenseNet network, which is better than RESNET network. It can be seen that the connections between its middle layers are very dense, and both layers are connected. This shows that the characteristics of each layer are shared and can be transmitted iteratively.

The upper layer in Figure 1(b) is a 12-layer denseness. The lower layer in Figure 1(b) is a 3-layer network structure, which represents the attention mechanism. Among them, C1 and C2 are two convolutional layers, *h* and *w* represent the size, F1 represents the convolution, F2 represents the squeeze operation, and the feature map is changed to a size of 1 through the convolution kernel, which has a global receptive field to some extent represents global distribution. F3 stands for excitation operation; it can update the weight. F4 represents the operation of scale to weigh the normalized weights to the features of each channel.

The attention model can learn deeper features. It consists of several small modules, including squeeze and exception. The squeeze operation is to obtain the global features, and then, the exception will learn the global features and then get the global weight, that is, the individual weight of each layer, and then, weigh the weight to the corresponding layer through operation. In fact, the attention mechanism represents that the layer with large contribution will highlight its characteristics, and the layer with small contribution will inhibit its characteristics.

The classification network of this paper also adopts the idea of integrated learning, which connects the DenseNet of the upper layer with the attention mechanism of the lower layer, which helps to improve the accuracy of the final network.

The target detection network uses the YOLO-V4 network, but there are inherent shortcomings in the application of the YOLO-V4 network to mask recognition. This defect comes from the inherent geometric structure of the module.

The convolution unit samples the fixed position of the input feature map; the pooling layer performs pooling at a fixed ratio; these characteristics have an impact on the research results. For example, in the same layer of convolution, the receptive fields of all activation units are the same. However, different positions may correspond to objects of different scales or deformations. Therefore, adapting to the scale or the size of the receptive field is required for precise positioning. The improvement of the YOLO-V4 network mainly focuses on the introduction of deformable convolution. Deformable convolution is shown in Figure 2(a).

As shown in the figure, the deformable convolution process is as follows.

After the input layer, there are two outputs. The first output can learn offset after a series of feature learning. After applying offset to the next output, the output structure is obtained. 2*n* of the first input in Figure 2 represents the offset in *X* and *Y* directions.

After deformable convolution, the output feature map is the feature map after translation.

The network used in this paper is shown in Figure 2(b), where Input represents the input image, BackBone network is the network proposed in this paper, Neck represents the target detection network inserted between BackBone and the last output layer, this paper represents FPN + PAN, and Output represents the output layer, which is divided into three outputs. Predict targets of different sizes.

By replacing the convolution in the original YOLO-V4 network with a deformable convolution, the network will automatically find the key areas of the mask during the model training process and will not convolve the unfocused areas due to the limitation of the convolution shape product.

## 4. Experimental Verification

This study uses the PyTorch deep learning framework; the training hyperparameters use YOLO-V4 hyperparameters and the public mask data set for training. To conduct comparative experiments, this study selected CenterNet, YOLO-V4, YOLO-V5 network, Internet network, YOLO-V3 network, and Mask R-CNN as a comparison group and finally got the result.

The dataset uses some common pictures of wearing masks.  Figure 3 shows some pictures of people wearing masks.

The data consisted of a total of 1927 photos, all of which were labeled with images downloaded from the Internet. In the course of training, 70% were used as the training set and 30% as the test set.

The labeling of the mask position in the dataset is not standard. The dataset used in this study is recalibrated by the label. The data after calibration are shown in Figure 4.

When training and improving the YOLO-V4 network, first train the reference network to wear a mask. Then, use the trained parameters as the initial parameters to improve the YOLO-V4 benchmark network. During training, batch sizes are set to 192. The initial learning rate is set to 0.01. Train for 600 epochs. The learning rate is changed every 100 epochs. The loss function used in training is the cross-entropy loss function:

(1) $$\begin{array}{c} C=-\frac{1}{n}\sum_{x}\left[y\;\ln\;a+\left(1-y\right)\ln\left(1-a\right)\right]. \end{array}$$

A phenomenon often encountered in network training is overfitting, which is caused by many reasons, such as too little data. This paper can alleviate this phenomenon by adding regularization to the loss function. Formula (2) adds L2 regularization, where *λ* is weight attenuation, and sets to 0.9:

(2) $$\begin{array}{c} L=C+\frac{\lambda }{2n}\sum_{w}w^{2}. \end{array}$$

Nonlinearity needs to be added between the network layers; otherwise, the deeper network is only equivalent to the shallow network. The well-known sigmoid function formula is as follows:

(3) $$\begin{array}{c} f\left(x\right)=\frac{1}{1-e^{-x}}, \end{array}$$

where *x* represents input and *f*(*x*) means output. According to formula (1), the output range is (0, 1), which is not a 0-centered distribution, which will cause the problem of gradient disappearance. Under normal circumstances, the sigmoid function will not be considered.

Formula (4) is the tanh function, which is relatively better than the sigmoid function:

(4) $$\begin{array}{c} f\left(x\right)=\frac{1-e^{-2x}}{1+e^{-2x}}. \end{array}$$

In which, the highest tanh function is 1 and the lowest is −1. Everything else is within this range. It can solve the problem of centralized distribution, but the disappearance of gradient is not solved because the output has upper and lower limits.

Equation (5) is a ReLU function that can solve the disappearance of gradient:

(5) $$\begin{array}{c} f\left(x\right)=\left\{\begin{array}{cc} x, & \left(x>0\right),\\ 0, & \left(x\leq 0\right), \end{array}\right. \end{array}$$

(6) $$\begin{array}{c} f\left(x\right)=\left\{\begin{array}{cc} \alpha \left(e^{x}-1\right), & \left(x<0\right),\\ x, & \left(x>0\right). \end{array}\right. \end{array}$$

When training and improving the YOLO-V4 network, first train the reference network to wear a mask. Then, use the trained parameters as the initial parameters to improve the YOLO-V4 benchmark network. During training, the batch sizes are set to 192, the initial learning rate is set to 0.01, the training is 600 epochs, and the learning rate is changed every 100 epochs. The accuracy and loss function curves during training are shown in Figures 5 and 6. After that, the calibrated dataset is used for network training.

The training uses the same RTX 2080Ti GPU for training; the single card, the number of iterations, and other parameters are the same. After training, mAP is selected as the evaluation standard to analyze and evaluate the network results.

Map is a commonly used evaluation standard in the target inspection model. It takes into account the accuracy and recall. It is a collection of the two. The higher the map, the better the performance of the model.

Table 1 represents the confusion matrix of classification results.

Among them, Positive example represents positive sample, Counterexample represents negative sample, Reality represents data, Forecast result represents forecast, TP and TN represent positive sample and negative sample with correct forecast, and FP and FN represent positive sample and negative sample with wrong forecast.

The formulas of recall rate and accuracy rate are shown in formulas (7) and (8):

(7) $$\begin{array}{c} R=\frac{\text{TP}}{\text{TP}+\text{FN}}, \end{array}$$

(8) $$\begin{array}{c} P=\frac{\text{TP}}{\text{TP}+\text{FP}}. \end{array}$$

Table 2 shows the specific values of the seven groups of models after training, including the AP value and mAP value of each category.

After many experiments, multiple values of *R* and *P* are obtained, and then, curves are obtained with *R* as abscissa and *P* as ordinate, and AP values are obtained by calculating the area of curves. Since there is only one category, AP is also a mAP.

The order of mAP size in the table is improved YOLO-V4, YOLO-V4, YOLO-V5, CenterNet, YOLO-V3, and Mask R-CNN.

The data in Table 2 show that the network proposed in this paper is the best network and suitable for the field of mask detection.

In addition to map, the target detection model also has the ROC curve, which defines false positive rate as *x*-axis and true positive rate as *y*-axis.

TPR: among all samples that are positive, the ratio of correctly judged positive is
  (9) $$\begin{array}{c} \text{TPR}=\frac{\text{TP}}{\text{TP}+\text{FN}}. \end{array}$$
FPR: among all the samples that are actually negative examples, the ratio of falsely judged positive examples is
  (10) $$\begin{array}{c} \text{FPR}=\frac{\text{FP}}{\text{FP}+\text{TN}}. \end{array}$$

The ROC curve can well reflect the performance of the model. Its area is AUC. The larger the AUC value, the better the model performance. The ROC curve is shown in Figure 7.

In order to test whether each improvement of the YOLO-V4 network is effective. This article did a second comparative experiment, followed by improved YOLO-V4; YOLO-V4 (hereinafter referred to as D-YOLO-V4) added to the improved DenseNet benchmark network, and YOLO-V4 (hereinafter referred to as T-YOLO-V4) network. The specific values after training include the AP value and mAP value of each category.

It can be seen from the figure that the ROC curve area of the six models in descending order is improved YOLO-V4, YOLO-V4, YOLO-V5, CenterNet, YOLO-V3, and Mask R–CNN. This result is consistent with the result obtained by the mAP evaluation system.

The order of mAP size in the table is improved YOLO-V4, T-YOLO-V4, D-YOLO-V4, and YOLO-V4.

It can be seen from Table 3 that the improved YOLO-V4 model has the best training effect, indicating that the network proposed in this article is suitable for mask target detection. The effect of D-YOLO-V4 and T-YOLO-V4 is better than that of YOLO-V4. It shows that the two improvements proposed in this article are effective. The effects of D-YOLO-V4 and T-YOLO-V4 are both worse than improving YOLO-V4, indicating that the idea of improving stacking in this article is correct and improving YOLO-V4 is the best. Its ROC curve is shown in Figure 8.

It can also be seen from the ROC curve that the ROC curve area from large to small is YOLO-V4, T-YOLO-V4, D-YOLO-V4, and YOLO-V4, which is basically consistent with the results obtained by the mAP evaluation system.

The improved YOLO-V4 network proposed in this article has verified its feasibility and accuracy through experiments and has great value in use. Improving the YOLO-V4 network can help better respond to face recognition with masks in the epidemic.

Although the accuracy of our method has reached the expected results, there are still many problems that have not been resolved. For example, the robustness of the algorithm is not good enough. The model studied in this article focuses on accuracy and is slightly lacking in speed. The next step is to increase its speed based on ensuring accuracy and consider actual deployment and use.

## 5. Conclusion

This paper proposes a mask recognition algorithm based on improved YOLO-V4 neural network and the integrated SE-Net and DenseNet network and introduces deformable convolution. Compared with other target detection networks, the improved YOLO-V4 neural network used in this paper improves the accuracy of face recognition and detection with masks to a certain extent.

## Figures and Tables

**Figure 1:** Schematic diagram of the classification network. (a) DenseNet network. (b) Join the attention mechanism DenseNet network.

**Figure 2:** Schematic diagram of the deformable convolution and improved YOLO-V4. (a) Schematic diagram of the deformable convolution. (b) improved YOLO-V4.

**Figure 3:** Some pictures in the dataset.

**Figure 4:** Part of the calibration picture in the dataset.

**Figure 5:** Accuracy curve of benchmark network.

**Figure 6:** Baseline network loss curve.

**Figure 7:** Network ROC curve.

**Figure 8:** ROC curve of the second experimental network.

**Table 1:** Confusion matrix of classification results.

Reality	Forecast result	
	Positive example (p)	Counterexample (N)
Positive example (P)	TP	FN
Counterexample (N)	FP	TN

**Table 2:** Results of each model.

	mAP
Improved YOLO-V4	0.913
YOLO-V4	0.901
YOLO-V5	0.872
CenterNet	0.881
YOLO-V3	0.842
Mask R-CNN	0.817

**Table 3:** The results of each model in the second group of comparative experiments.

Methods	mAP
Improved YOLO-V4	0.913
D-YOLO-V4	0.903
T-YOLO-V4	0.907
YOLO-V4	0.901

## Data Availability

The simulation experiment data used to support the findings of this study are available from the corresponding author upon request.
